The article "Bloom's Classification of Educational Objectives Based on Deep Learning Theory Teaching Design of Nursing Specialty" was retracted in 2023. Reasons: signs of a paper mill; compromised peer review; unreliable results or conclusions.

# Bloom's Classification of Educational Objectives Based on Deep Learning Theory Teaching Design of Nursing Specialty

**DOI:** 10.1155/2022/3324477

**Published:** 2022-07-21

**Authors:** Jia zheng, Jarrent Tayag, Yingai Cui, Jiajun Chen

**Affiliations:** ^1^Angeles University Foundation, MacArthur Hwy, Angeles 2009, Pampanga, Philippines; ^2^Guangdong Medical University, College of Nursing, Dongguan 523808, Guangdong, China; ^3^Philippine Women's University, Manila 1004, Philippines

## Abstract

Through the effective integration of various teaching resources, carry out the teaching design of “basic nursing technology” for the nursing specialty in the information environment based on Bloom's education objective classification. Select 200 nursing students from two natural classes in the third year of undergraduate nursing major as the research objects with100 students in the experimental group and 100 students in the control group. The experimental group adopted Bloom's objective classification teaching mode, and the control group adopted the traditional teaching model. They have carried out the teaching intervention to ensure the consistency of teachers, textbook use, teaching hours, and teaching progress between the two groups. The evaluation model of the teaching design results is the RBF neural network. The model improves the convergence ability of the RBF network by dynamically changing the control parameters of the L-M algorithm. RBF realizes the goal of the comprehensive analysis of course teaching effects evaluation and various influencing factors. The results showed that the differences in self-management ability, information ability, cooperation score, and total score of the experimental group were significantly higher than those of the control group, with statistical significance (*P* < 0.01). The teaching of Bloom's educational objective model can enhance students' subjective consciousness and effectively improve their independent learning ability. The learning effect is improved obviously. This paper studies the teaching approaches to improve nursing students' comprehensive ability and humanistic care quality and provides a reference for deepening nursing undergraduate teaching reform.

## 1. Introduction

Essential Nursing Technology is based on primary and clinical medicine and integrates humanistic management and other disciplines. The nursing staff must have rich theoretical knowledge and comprehensive solid nursing skills for internal medicine diseases involving various ages and complex and changeable conditions [1]. Clinical practice can provide a good platform for nursing students to apply theoretical knowledge and essential links to acquire perceptual and rational expertise and experience. Throughout the current situation of nursing education in China, students are in a passive learning state, mechanical imitation, and rote memorization, weakening students' comprehensive quality and skills. The problem is that the traditional teaching concept is deeply rooted. Theoretical teaching still occupies a large proportion. The practical learning stage in the last year of nursing students and the academic learning stage in the early stages are prolonged. The practical training and probation courses during the school hours are more miniature and do not reach the standard teaching objectives. However, some developed foreign countries attach great importance to the cultivation of nursing students' comprehensive ability, the education concept's advances, and the alternating combination of “theory and practice” in teaching, cultivating many applied nursing talents adapted to modern medical treatment. Therefore, narrowing the gap with foreign developed countries, breaking the traditional teaching method of thinking set, and deepening the reform of nursing teaching has become a significant challenge facing most nursing educators [2].

Bloom's theory of classification of educational objectives is the earliest analytical tool for evaluating classroom teaching purposes. Behaviorism is the foundation of Moding's analytical tool. Bloom's goal classification theory originated from a research team led by Bloom that proposed a goal classification framework for college examiners and evaluators [3]. Bloom's goal classification theory has significantly influenced education. The cognitive goal classification method has played an important role up to now. According to students' different levels of cognition, the theory divides the goal of cognitive dimension into six classes: memorization, understanding, application, analysis, synthesis, and evaluation. But the original bloom theory did not illustrate how to apply knowledge to practice [4]. The results of later version of the revision will be in the field of cognitive learning. They are divided into four categories: factual knowledge, conceptual knowledge, procedural knowledge, and metacognitive knowledge. At the same time, you will get the results of the study process divided into six levels; from low to high: Remember, understand, apply, analyze, evaluate and create [5].

The concept and development of nursing practice teaching in foreign countries are based on application, focusing on strengthening students' practical ability training. Practice education runs through the whole process of nursing talent training in universities, advocating students' early contact with clinical practice [6]. Research shows that foreign universities pay special attention to the form of “bedside teaching” to cultivate students' clinical practice ability and clinical thinking ability in clinical practice teaching. There are many hours of practical training, probation, and internship, and the teaching mode of clinical practice and theoretical learning is simultaneous. The “institutionalization concept” of practical foreign education establishes the development direction of university education, which combines knowledge and training, understanding and thinking, classroom and outside, and theory and experience [7]. It provides an ideological and institutional guarantee for universities to improve their talents' innovative ability, practical ability, and collaboration ability. China and Japan have the same nursing practice teaching mode, and both adopt the full practice mode. However, nursing students in Japan must go back to school after the 8-month graduation and learn theoretical knowledge again, focusing more on the combination of clinical and basic, clinical and social. In contrast, China's nursing undergraduate practice curriculum only focuses on clinical [8]. In comparison, Japan's nursing clinical practice curriculum arrangement is more scientific and reasonable. The seamless connection with clinical practice enables students to grasp the theoretical knowledge more firmly and ensures the practicality and comprehensiveness of talent training [9]. Many literature studies have shown that the significant difference between nursing education in western developed countries and nursing education in China lies in the setting of practical courses. Foreign higher medical universities to each nursing professional class time to arrange a lot of clinical practice, and clinical practice in the teaching, formed a kind of full nursing practice teaching mode. This scheme exercises nursing students' clinical skills, innovation, communication, and comprehensive analysis and solves a large number of literature. The significant difference lies in the setting of practical courses between western and Chinese culture.

Based on the above research, so many reviews, and a complete investigation, this article closely focused on the new “Internet+” education reform trend. For “basic nursing technology,” design and implement teaching designs based on deep learning theory from the perspective of Bloom's classification of educational objectives. In evaluating teaching design results, the RBF neural network model is innovatively used to train, verify, process, and maintain the teaching design results. Introduced the advantages of the RBF neural network in the teaching quality evaluation system in colleges and universities, which makes the quality evaluation systematic, quantitative, and objective. In all 100 test samples, the RBF network achieved 92% accuracy in evaluation. Evaluation results show the bloom education of primary nursing technology teaching has changed the traditional teaching model. The students' work in simulated situations can improve their skill level and theoretical knowledge. This method improves students' independent learning and critical thinking abilities and stimulates students' learning interests and initiative, promote the effective combination and synchronous development of professional theoretical knowledge and practical skills. Strengthen students' sense of identity in hospital culture and the nursing profession; expand new ways of collaborative education among colleges and universities to achieve the training goal of high-quality applied nursing talents.

## 2. Teaching Design Based on Bloom Education

### 2.1. Teaching Objective Design

Establishing curriculum teaching objectives is the starting point and key to teaching design and the principal basis of teaching quality inspection and evaluation. The establishment of teaching objectives for project-based courses should reflect the requirements of the occupation, including vocational ability objectives and corresponding knowledge objectives. Among them, based on the vocational ability goal, the role, and task of the course, in-depth vocational job research, and reference to the actual situation of students and majors, the determination of the knowledge goal is based on the vocational ability goal, to be “necessary, enough” [10]. The primary nursing technology is a basic introductory course, nursing learning areas of nursing jobs through in-depth research, combined with the teaching outline and the exam outline requirements. According to professional ability, method ability, and social ability, three aspects division to develop the introductory nursing technology course's overall goal, Table 1. Then, according to Bloom's education theory, specific teaching objectives are formulated for each project according to knowledge objectives, ability objectives, and quality objectives.

### 2.2. Teaching Content Design

Based on experience and the skilled jobs and tasks for further research, analysis of education experts and nurse specialists in three armor hospitals were needed for the final engaged in practical vocational ability and to complete the specific work tasks [11]. Basic nursing is divided into four extensive teachings based on clinical work and 15 practice projects, breaking the pattern of traditional schooling. The work process serves as the guide. Education is a teaching base integrating science and practice, aiming to make the cultivated students meet the requirements of the related vocational posts in this course and realize the close connection between talent training and post needs. Tables 2 and 3 show specific items.

It notes that because students do not have working experience and the ability to complete some projects independently, we will design the project again based on some complicated project implementation to make it suitable for learners [12]. Drug administration projects include iv infusion, oral drug administration, atomization inhalation, intramuscular injection, subcutaneous injection, intradermal injection, and drug allergy tests [13]. The rescue projects for critically ill patients were divided into intravenous blood transfusion, gastric lavage, oxygen inhalation, sputum aspiration, and cardiopulmonary resuscitation. And then integrate to cultivate students' ability to do things and global awareness [14].

### 2.3. Unit Instructional Design

The overall curriculum design is to solve the problem of how to do a good course, and the unit design is to solve the problem of how to do a good lesson. Each class can effectively guide students to form the corresponding professional ability. In unit teaching design, the following three aspects need to be paid attention to:[15].

1. Take students as the center, stimulate students' learning interests and motivation, and have teachers mainly play the roles of guidance, coordination, and assessment in class.
2. The integration of “teaching, learning, and doing” enables students to learn by doing and acquire skills and corresponding theoretical knowledge.
3. Attach importance to unit assessment. To promote learning through assessment, students assess and evaluate after completing each project task to mobilize their enthusiasm and motivation. The unit design includes the preparation stage and implementation stage, as follows:

Implementation of the project teaching process is the most important and most complex phase, and it is difficult for students without experience. To improve the learning effect, introducing this link added some teaching steps in the project, including the project's comprehensive explanation, demonstration, and operation concept explanation [16]. The project comes to its implementation, and students will focus on learning again according to the specific situation. For example, when finding some common problems or difficulties, the teacher will arrange a time to explain them to ensure the smooth progress of the project.  Table 4 shows the specific teaching process.

## 3. Teaching Evaluation Design Based on RBF Neural Network

The RBF network proves to approach any nonlinear type function and deal with the regularity challenges in the system. It has outstanding generalization ability and an obvious convergence speed advantage and applies successfully to many fields such as time series analysis, nonlinear function approximation, pattern recognition, data classification, image processing, information processing, fault analysis, system modeling, and intelligent control[17].

### 3.1. RBF Neural Network Structure

The structure of the multilayer forward network is similar to that of the RBF network [18]. The RBF network is also a forward network, which has three layers. The signal source node constitutes the input layer; the hidden layer is the second layer. Determine the number of hidden elements according to the situation of the problem to be described. The remote part adopts the RBF radial basis transformation function, and the third layer is the linear output layer.  Figure 1 shows the topology of the RBF network.

The RBF neural network is suitable for solving classification and evaluation problems. It belongs to a forward neural network approximating any continuous function with precision.

Classification is a particular case of approximation, which is classification generalization. When each type of sample is one, that is, when all instances are separately classified, the classification problem is an approximation problem.

According to the RBF interpolation principle, the number of nodes in the network's hidden layer is the number of samples, which makes the network structure directly related to the problem size. When there are too many samples, the approximation ability is not ideal. For classification problems, the number of hidden layer nodes can equal the number of sample classes. In this case, RBF can improve the network performance significantly.

### 3.2. RBF Neural Network Model

As for the determination method of the RBF network model, input nodes and output nodes are determined according to specific problems to be solved. The number of input nodes is the number of influencing factors, while the number of output nodes is the number of grades of evaluation results [19]. Clustering algorithms or multiple experiments usually determine hidden layer nodes. Let the input layer consist of N nodes, the hidden layer of H nodes, and the output layer of *M* nodes.  Figure 2 shows the network model.

The characteristic of this model is to fix the hidden layer weight. *w*_*ij*_ is always 1. The hidden layer excitation function is the Gaussian function. The output layer is a linear combination of the hidden layer outputs. Network parameters are the center *c*_*j*_ of each node in the hidden layer and variance *σ*_*j*_^2^; output weight *v*_*jk*_. The input-output relation of the model is as follows:

(1) $$\begin{array}{c} y_{k}=\sum_{j=1}^{k}v_{jk}\exp\left(-\frac{{\left\|x-c_{j}\right\|}^{2}}{2\sigma_{j}^{2}}\right). \end{array}$$

### 3.3. RBF Neural Network Algorithm

#### 3.3.1. RBF of Fixed Center

Network parameters are output layer weights only. A clustering algorithm can determine the centers (K-means clustering algorithm). Empirical formulas $\sigma^{2}=d\max/\sqrt{h}$ and *d*max can evaluate the maximum Euclidean distance between centers, and *h* is the number of centers *V*_*h*_. In this case, the weight of the output layer can be directly solved by linear equations without iteration, thus significantly improving the learning speed. Let *T* and *Y* represent the expected output and actual output of the sample, respectively; Φ is the output of the RBF function of the hidden layer, and the output layer calculates the weight as follows:

(2) $$\begin{array}{c} E=\frac{1}{2}{\left(T-Y\right)}^{T}\left(T-Y\right)\\ =\frac{1}{2}{\left(T-\Phi V\right)}^{T}\left(T-\Phi V\right)\\ =\frac{1}{2}\left(T^{2}T-2T^{T}\Phi V+V^{T}\Phi^{T}\Phi V\right). \end{array}$$

Equations (2) is a linear system of equations about the weights of the output layer. When the number of samples is large (more than the number of importance), the system is contradictory with no exact solution. In this case, the equation uses the least square method to transform it into a regular plan.

(3) $$\begin{array}{c} \frac{\partial E}{\partial V}=0\Rightarrow -\Phi^{T}T+\Phi^{T}\Phi V\\ =0\Rightarrow V={\left(\Phi^{T}\Phi \right)}^{-1}\Phi^{T}T. \end{array}$$

For the normal equations (3), Jacobian substitution method or Gauss–seidel iterative method can be used to solve.

#### 3.3.2. RBF of Gradient Descent

The calculation used the BP algorithm to simultaneously train the center, variance, and output layer weights of hidden layer RBF neurons.

(4) $$\begin{array}{c} \text{Let the input sample be}:\left\{X^{1},X^{2},\ldots ,X^{P}\right\},X^{k}=\left(x_{1}^{k},x_{2}^{k},\ldots ,x_{n}^{k}\right),\\ \text{The output sample is}:\left\{D^{1},D^{2},\ldots ,D^{P}\right\},D^{k}=\left(d_{1}^{k},d_{2}^{k},\ldots ,d_{m}^{k}\right) \end{array}$$

The hidden layer output is: *q*_*i*_=exp(−‖*X* − *c*_*i*_‖^2^/*σ*_*i*_^2^), the network output is: *y*_*k*_=∑_*i*=1_^*h*^*w*_*ik*_*q*_*i*_

The error function is: *J*=1/2∑_*p*=1_^*p*^‖*d*^*p*^ − *y*^*p*^‖^2^, according to the gradient descent method, the gradient calculation formula of parameters of each layer is as follows:

(5) $$\begin{array}{c} \frac{\partial J}{\partial v_{ik}}=-\sum_{p=1}^{p}\sum_{k=1}^{m}\left(d_{k}^{p}-y_{k}^{p}\right)q_{i}^{p},\\ \frac{\partial J}{\partial c_{i}}=-2\sum_{p=1}^{p}\sum_{k=1}^{m}\left(d_{k}^{p}-y_{k}^{p}\right)w_{ik}q_{k}^{p}\left(\frac{X^{p}-c_{i}}{\sigma_{i}^{2}}\right),\\ \frac{\partial J}{\partial \sigma_{i}}=-2\sum_{p=1}^{p}\sum_{k=1}^{m}\left(d_{k}^{p}-y_{k}^{p}\right)w_{ik}q_{k}^{p}\frac{{\left(X^{p}-c_{i}\right)}^{2}}{\sigma_{i}^{3}}. \end{array}$$

The specific adjustment method is as follows: *v*_*ik*_=*v*_*ik*_ − *α*(*∂J*/*∂v*_*ik*_), *c*_*i*_=*c*_*i*_ − *α*(*∂J*/*∂c*_*i*_), *σ*_*i*_=*σ*_*i*_ − *α*(*∂J*/*∂σ*_*i*_)

### 3.4. Evaluation Results and Analysis

This paper obtains the input data for information collection by using the method of students' online evaluation of teaching. That is to input the indicators in the student evaluation table into the classroom teaching quality evaluation system and then organize students to score and evaluate the course. Students can complete the evaluation independently in the online assessment process. In addition, to assessing the score, students can also express their own opinions or opinions about the course. The evaluation online has the following challenges: time and space, interactivity, openness, the spread of sex, convenience of data collection management, personalized communication, and convenient data statistics and analysis functions. This way becomes the mainstream of the current university's information acquisition and introduces the advantage of the network classroom teaching quality evaluation system. The quality evaluation has realized systematization, quantification, and objectification.

Five hundred thirty samples of data from five design processes were submitted to the RBF network for training to approximate the complex mapping relationship between evaluation indexes and various evaluation results. The network converges after 3385 iterations.  Figure 3 shows the dynamic curve of approximation error decreases with the number of iterative steps.

Since the network's output is real, it is necessary to transform the quantitative numerical results into qualitative evaluation grades. Let the numerical result of the *i* sample output be Y. According to Table 4.1, if *y*, <0.59 is unqualified, 0.60 < *y* < 0.69 is qualified, 0.70 < *y* < 0.79 is medium, 0.80 < *y* < 0.89 is good, and 0.90 < *y* < 1.00 is excellent. According to the scheme designed above, Table 5 shows the training results of some samples.

In all 100 test samples, the maximum test error is 0.0513. 92 models are correct, seven pieces are excellent, and the remaining three specimens are medium. Therefore, the evaluation accuracy rate of the RBF network is as high as 92%. The verification results show that the RBF neural network and the evaluation model of the course teaching effect have strong generalization ability. It is a feasible and reasonable evaluation model which provides a new way to solve the comprehensive evaluation problem of the teaching effect in colleges and universities.

Select the traditional teaching model control group and the new teaching mode experimental group for comparative analysis of teaching quality.  Table 6 is the evaluation result.

Table 6 shows that the differences in self-management ability, information ability, combination score, and total score of the experimental group were significantly higher than those of the control group, with statistical significance (*P* < 0.01). The teaching of Bloom's educational objective model can enhance students' subjective consciousness and effectively improve their independent learning ability. The learning effect is improved obviously.

## 4. Conclusion

Bloom education target classification under the perspective of “basic nursing technology project,” the implementation of teaching design has changed the traditional teaching model. Bloom education orients the working process with a project as the carrier, lets the student more in line with the cognitive learning and skill formation of the situation, fully mobilizes, and excavates the students' potential, and improves the students' skills and theoretical knowledge. It improves students' independent learning abilities and critical thinking abilities and stimulates students' interest and initiative in learning. Obtain the following conclusions:

1. Bloom's taxonomy of educational objectives can reveal the depth levels of students' teaching effects by employing students' behaviors and using bloom's taxonomy of educational purposes to design the teaching of essential nursing technology for nursing majors.
2. Study the mapping mechanism and training method of the RBF network, propose the evaluation model of RBF teaching effect based on the L-M algorithm, and give the model establishment method, sample selection method, and network training method in detail. Experimental results show the validity of the model. The establishment of this model provides a new way to evaluate the teaching effect objectively and impartially.
3. The teaching effects of different teaching modes in the experimental and control groups were compared and analyzed. The differences in self-management ability, information ability, cooperation score, and total score of the experimental group were significantly higher than those of the control group, with statistical significance (*P* < 0.01). Bloom's educational objective teaching mode can enhance students' subjective consciousness and effectively improve their independent learning ability. The learning effect is improved obviously.

## Figures and Tables

**Figure 1:** Topology of the RBF network.

**Figure 2:** RBF neural network model.

**Figure 3:** Decrease curve of approximation error in RBF training process.

**Table 1:** Teaching objectives of Basic Nursing Technology.

Ability	Instructional objectives
Professional competence	Master the basic theory and knowledge of basic nursing technology;
	Master the basic nursing operation techniques of each standard;
	The ability to correctly implement various nursing techniques and evaluate their effects according to the changes in patients' conditions;
	Ability to process medical orders and related medical documents timely and accurately;
	The ability of observation, emergency treatment and rescue cooperation for acute and critically ill patients.

Methods ability	Have particular self-study ability, understanding ability, and expression ability;
	Good ability to acquire, analyze, summarize, absorb and use new knowledge;
	Ability to combine and transfer theoretical knowledge with clinical practice;
	Good critical thinking ability.

Social competence	Have good professional sentiment, professional ethics, and professional quality;
	Good communication, coordination, and cooperation skills;
	Reasonable psychological adjustment and social adaptability;
	Strong sense of responsibility;
	He has the spirit of humanitarianism and conscientiousness.

**Table 2:** Teaching content of patient admission nursing.

Workflow	Practice project	Project tasks	Period
Admission of new patients	Outpatient/emergency care	Outpatient nursing/emergency nursing work	4
	Outpatient (emergency patient inpatient care	Bed preparation unit	2
		Admission of new patients	2
		Measurement of vital signs	2
		Record medical records and nursing records	3
		To deal with the doctor's advice	3
		Grading nursing	2
		Safety nursing	2
		The implementation of the diet	2
	Prevention and control of infection	Cleaning, disinfection, sterilization, hand hygiene, aseptic technology, isolation technology in the ward	18

Patient discharge care	Discharge	Nursing of discharged patients	2
		Process medical care documentation	1
		Deal with ward and bed units	1

**Table 3:** Nursing teaching contents of patients during hospitalization.

Workflow	Practice project	Project tasks	Period
Specimen collection	Specimen collection	Morning/emergency specimen collection	6
Sanitation and hygiene	Sanitation and hygiene	Mouth care	4
		Facial cleanses and hair treatments	4
		Skin care	4
	Morning care	Bed making unit	2
		Patients change bed units	3
		Position and change lying position	2

Care	Dispensing drugs	Drug allergy test	6
		Parenteral administration	6
		Venous transfusion	6
		Oral medication	6
		Aerosolization	6
		Local drug delivery	6

Diet nursing	Diet nursing	Assess nutritional status	4
		General patient diet nursing	4
		Dietary nursing for special patients	4

Discharge care	Urine and feces assessment and care	Assess urine and feces	6
		Nursing of abnormal urination and defecation	6

Comfortable nursing	Comfortable nursing	Guide rest and activity	4
		Assess and care for pain	4

Night nursing	Night nursing	Bed making unit	2
		Perineum nursing	2
		Sleep care	2

Care of critically ill patients	Disease observation	Observation and nursing of critically ill patients	2
		Vital signs observation and nursing (including cold and heat treatment)	2
		Consciousness, pupil, general observation	2
		Record intensive care records	2
		Supportive care for critically ill patients	2

Cooperate with doctors in rescue work	Rescue of critically ill patients	Iv blood transfusion, gastric lavage, oxygen inhalation, sputum aspiration, cardiopulmonary resuscitation	14
		Use of artificial breathing apparatus	6

Hospic care	Hospic care	Physical and mental care for terminal patients	4
		Body care	2

**Table 4:** The teaching process of Bloom's classification of educational objectives.

Teaching link	Teaching process design
Project introduction	Assign project assignments, and provide teaching videos and teaching materials. The first class introduces the project and shows examples. The teacher will explain the theoretical content of the project and the project's objectives and quality requirements and demonstrate the project's specific process and operation methods through role-playing and other teaching methods.
Project scheduling	Team members will discuss and make project plans according to project tasks, including goal setting, scenario design, material preparation, role division, workflow, and time control. Teachers will give operational guidance in this process.
Project implementation	Open the training room, and set up the clinical work situation, according to the project tasks equipped with relevant operation materials; according to the project task book and plan, students complete the project tasks. They can consciously develop a sense of teamwork based on the study, train their skills in completing the job, and understand and memorize relevant knowledge. Teachers provide timely guidance and explanation, correct students' mistakes at any time, and explain common problems in completing project tasks. Teachers provide timely advice and reason, right students' mistakes at any time, and explain common problems in completing project tasks.
Achievement exhibition	Students in each group show their project results (including videos and documents) on the network platform. Carry out teacher evaluation, expert evaluation, group evaluation, and self-evaluation, arrange excellent project results, and provide a platform for students to show their style.
Evaluation summary	Guide the students to summarize the learning achievements, and then the teacher comments on the summary. Finally, teachers carried out the project unit assessment, and each group submitted a project report for evaluation. Let's move on to the next project.

**Table 5:** Training results of some samples.

Group	Serial number	The actual output	Desired output	The training results	Experts results
Experimental group	1	0.9581	0.95	Excellent	Excellent
	2	0.9569	0.95	Excellent	Excellent
	3	0.9467	0.95	Excellent	Excellent
	……	……	……	……	……
	100	0.9488	0.95	Excellent	Excellent

Control group	1	0.8551	0.85	Well	Well
	2	0.8577	0.85	Well	Well
	3	0.8537	0.85	Well	Well
	……	……	……	……	……
	100	0.85121	0.85	Well	Well

**Table 6:** Variation analysis.

	Experimental group	Control group	*t*	*P*
Self-management ability	6.9 ± 2.4	1.6 ± 2.9	11.015	<0.01
Information ability	6.7 ± 2.8	-1.7 ± 3.4	15.194	<0.01
Ability to cooperate	4.1 ± 2.2	0.7 ± 2.9	7.528	<0.01
Total score of independent learning ability	17.6 ± 4.0	3.7 ± 4.3	17.703	<0.01

## Data Availability

The dataset used in this study is available upon reasonable request.
